The article "Comparison of choroidal thickness measurements using swept source and spectral domain optical coherence tomography in pachychoroid diseases" was published in 2020. Journal: PLoS One.

# Comparison of choroidal thickness measurements using swept source and spectral domain optical coherence tomography in pachychoroid diseases

**DOI:** 10.1371/journal.pone.0229134

**Published:** 2020-02-26

**Authors:** Min-Woo Lee, Hye-Jin Park, Yong-Il Shin, Woo-Hyuk Lee, Hyung-Bin Lim, Jung-Yeul Kim

**Affiliations:** 1 Department of Ophthalmology, Konyang University College of Medicine, Daejeon, Republic of Korea; 2 Department of Ophthalmology, Chungnam National University College of Medicine, Daejeon, Republic of Korea; Nicolaus Copernicus University, POLAND

## Abstract

**Purpose:**

To determine the comparability of choroidal thickness (ChT) measurements using swept source (SS) and spectral domain (SD) optical coherence tomography (OCT) devices in patients with pachychoroid diseases.

**Methods:**

Patients with pachychoroid diseases were recruited. OCT scans were performed sequentially with a Cirrus HD OCT 5000 and Plex Elite 9000. Images were analyzed by two independent observers. Each image was independently measured twice by each observer to determine the intraobserver repeatability.

**Results:**

A total of 55 eyes were included. The average ChT of the subfoveal area using SS-OCT and SD-OCT was 430.5 ± 68.1 and 428.5 ± 57.9 μm, respectively, which did not show a significant result as the main effect in the repeated-measure analysis of variance (P = 0.067). Using SS-OCT, the intraobserver intraclass correlation coefficient (ICC) of both observers was > 0.950 at every measured point, and the interobserver coefficient of repeatability (CR) of the subfoveal area was 45.1 μm (95% confidence interval (CI), 40.8–49.4). Using SD-OCT, the intraobserver ICC of both observers was > 0.800, and the interobserver CR of the subfoveal area was 71.2 μm (95% CI, 64.4–78.0). Additionally, the intraobserver and interobserver CRs showed significantly better repeatability in SS-OCT than SD-OCT in F-test. In patients with ChT ≥ 400 μm, the interobserver CRs of SS-OCT and SD-OCT were 48.4 (95% CI, 42.6–54.2) and 95.2 μm (95% CI, 83.9–106.6), respectively. In patients with a subfoveal active lesion, the interobserver CRs were 44.5 (95% CI, 37.6–51.4) and 100.1 μm (95% CI, 84.6–115.5), respectively.

**Conclusions:**

Although the ChT measurements were comparable between SS-OCT and SD-OCT devices in pachychoroid diseases, SD-OCT showed low reliability in patients with ChT ≥ 400 μm and subfoveal active lesions. SS-OCT would be therefore more suitable for observation and follow-up of choroidal structures in pachychoroid diseases.

## Introduction

The term pachychoroid has been used widely in recent studies. The pachychoroid spectrum diseases, including pachychoroid pigment epitheliopathy (PPE), central serous chorioretinopathy (CSC), pachychoroid neovasculopathy (PNV), and polypoidal choroidal vasculopathy (PCV), are thought to underlie the development of focal disruptions in the retinal pigment epithelium (RPE) and Bruch’s membrane, leading eventually to various clinical manifestations.[1, 2] The phenotype of these diseases is characterized by diffuse or focal areas of increased choroidal thickness (ChT), dilated choroidal vessels, and structural changes according to optical coherence tomography (OCT) with thinned choriocapillaris and Sattler’s layer overlying the pachyvessels.[1–4] Therefore, it is critical to observe the structure of the choroid in pachychoroid diseases.

OCT technology has recently made remarkable process, and development of enhanced depth imaging (EDI) has improved the image quality of deeper structures.[5] Swept-source OCT (SS-OCT) especially enables the choroid to be imaged at greater depth and using shorter acquisition times than those required for EDI using spectral-domain OCT (SD-OCT).[6] So many previous studies have reported the analysis of ChT or choroidal images using these two devices.[6–9] Tan et al.[7] reported that subfoveal ChT measurements were comparable between the two devices, and the presence of retinal disease increased the variability of ChT measurements between the OCT devices. Waldstein et al.[6] reported that both SD-OCT using EDI/frame averaging and SS-OCT provided excellent visualization capabilities for volumetric imaging of the choroidoscleral interface. However, to the best of our knowledge, no comparison of ChT measurements using SS-OCT and SD-OCT in patients with pachychoroid diseases has been reported.

The purpose of this study was to determine the comparability of ChT measurements using SS-OCT and SD-OCT in the pachychoroid, and to evaluate potential factors affecting the reliability of the measurements.

## Methods

### Patients

This study adhered to the tenets of the Declaration of Helsinki and was approved by the Institutional Review Board of Chungnam National University Hospital in the Republic of Korea. Patients who visited our retinal clinic from June 2018 to February 2019 were analyzed retrospectively, and patients with pachychoroid diseases such as PCV, CSC, PNV, and PPE were recruited for the study. The requirement for obtaining informed patient consent was waived due to the retrospective nature of the study. Patients who had any intraocular surgery except cataract surgery were excluded. A detailed history, best-corrected visual acuity (BCVA), intraocular pressure using non-contact tonometry, spherical equivalent, and axial length using an IOL Master (Carl Zeiss, Jena, Germany) were determined. Patients were imaged using both SD-OCT and SS-OCT with a 5-min interval between measurements.

### OCT imaging

SD-OCT images were obtained using the Cirrus HD OCT 5000 (Carl Zeiss Meditech, Dublin, CA; version 10.0), which has an axial resolution of 5 μm and lateral resolution as 15 μm. HD 1 line 100× scan generates a single high definition scan at a depth of 2.0 mm with 100 B-scans, each composed of 1024 A-scans. The line length of the scan was adjusted to 9 mm.

SS-OCT images were obtained using the Plex Elite 9000 (Carl Zeiss Meditech, Dublin, CA; version 1.50), which has an axial resoultion as 1.95 μm and lateral resoultion as 20 μm. HD spotlight 1 (10–100×) scan generates a single high definition scan at a depth of 3.0 mm with 100 B-scans, each composed of 1024 A-scans. The length of the scan was adjusted to 9 mm as in the SD-OCT images.

All images were obtained using the EDI mode, and images with a signal strength < 7 were excluded.

### Choroidal thickeness measurements

The ChT was measured as the perpendicular distance from the outer portion of the hyperreflective line corresponding to the retinal pigment epithelium to the posterior edge of the choroid as demarcated by the hyperreflective line corresponding to the chorioscleral interface as previous studies using software calipers at five points: the subfoveal area, and at the temporal and nasal points at radii of 500 and 1500 μm (Fig 1).[10–12] The foveal center, defined as subfoveal area, was confirmed by comparing orientation of the HD scan to the 5-line raster OCT scan as the previous study.[10] The pachyvessel diameter (vertical diameter of the thickest outer choroidal vessel in the foveal region) was also measured using software calipers, and choroidal caverns were identified as focal hyporeflective spaces on B-scan images from 2 devices.

**Fig 1:** Choroidal thickness, pachyvessel diameter, and choroidal cavern (red arrows) on swept source (SS) and spectral domain (SD) optical coherence tomography (OCT) images. Chroidal thickness was obtained by measuring the perpendicular distance from the outer portion of the hyperreflective line corresponding to the retinal pigment epithelium to the inner surface of the sclera using software calipers at five points: the subfoveal area, and at the temporal and nasal points at radii of 500 and 1500 μm.

The images were analyzed by two independent observers (M.W.L. and H.J.P.) who were blinded to each other’s measurements and their previous measurements. Each image was independently measured two times by each of the two observers to analyze intraobserver repeatability.

### Statistical analyses

A repeated-measure analysis of variance (ANOVA) was performed using 4 within-subjects factors of OCT device, observer, order of measurement, and measurement location. The average values of the two observers were used to compare measurements of the two different devices. The agreement between intraobserver and interobserver measurements for each SD-OCT and SS-OCT device was assessed using the coefficient of repeatability (CR), intraclass correlation coefficient (ICC), and Bland-Altman plots. The 95% confidence intervals for the upper and lower limits of agreement in the Bland-Altman graphs were calculated as follow; for the upper limits of agreement, mean of the difference (*d*) + coefficients_0.025_·standard deviation (*S*) and *d* + coeffeicnts_0.975_·*S*; for the lower limits of agreement, *d*—coefficients_0.025_·*S* and *d*—coeffeicnts_0.975_·*S*.[13] The CR was calculated using the method described by Bland-Altman as 2.77 S_W_ (within-subject standard deviation).[14] An ICC, the ratio of the subject variance to the total variance, close to 1 means that the variance is low in the same examination (< 0.40, poor; between 0.40 and 0.59, fair; between 0.60 and 0.74, good; between 0.75 and 1.00, excellent). Intraobserver and interobserver repeatabilities of choroidal thickness measurements were further compared using the F-test. Statistical analyses were performed using SPSS software for Windows, version 18.0 (IBM Corp., Armonk, NY).

## Results

Among 67 eyes, 2 cases (3.2%) in SS-OCT images and 12 cases (17.9%) in SD-OCT images were excluded because of the invisible posterior boundary. As a result, a total of 55 eyes in which the choroidal boundaries were identified using both SD- and SS-OCT instruments were included in the study: 18 eyes with CSC, 10 eyes with PCV, 5 eyes with PNV, and 22 eyes with PPE (Table 1).

**Table 1:** Demographics and baseline characteristics of patients.

Number of eyes	55
CSC	18 (32.7%)
PCV	10 (18.2%)
PNV	5 (9.1%)
PPE	22 (40%)
Age, years (range)	51.2 ± 15.9 (19–81)
Sex (male, n)	38 (69.10%)
Laterality (right, n)	30 (54.5%)
BCVA, logMAR (range)	0.09 ± 0.25 (-0.18–1.30)
Spherical equivalent, diopters (range)	-0.12 ± 1.65 (-6.75 - +4.00)
IOP, mmHg (range)	15.3 ± 2.5 (10–20)
Axial length, mm (range)	23.4 ± 0.8 (21.1–25.5)
Mean CMT, μm (range)	257.7 ± 75.4 (152–571)

CSC, central serous chorioretinopathy; PCV, polypoidal choroidal vasculopathy; PNV, pachychoroid vasculopathy; PPE, pachychoroid pigment epitheliopathy; SD, standard deviation; BCVA, best-corrected visual acuity; IOP, intraocular pressure; CMT, central macular thickness

The mean age was 51.2 ± 15.9 years, the mean BCVA was 0.09 ± 0.25, the mean axial length was 23.4 ± 0.8 mm, and the mean central macular thickness (CMT) was 257.7 ± 75.4 μm.

### ChT measurements using the two different devices

The average ChTs of the subfoveal area between the two observers using SS-OCT and SD-OCT were 430.5 ± 68.1 μm (range, 300 to 645 μm) and 428.5 ± 57.9 μm (range, 293.5 to 606 μm), respectively (Table 2).

**Table 2:** Choroidal thickness measurements using swept source (SS) and spectral domain (SD) optical coherence tomography (OCT).

	Average SS	Average SD
Subfoveal	430.5 ± 68.1	428.5 ± 57.9
Temporal 500 μm	407.8 ± 82.5	409.1 ± 69.2
Temporal 1500 μm	378.5 ± 87.0	378.3 ± 77.6
Nasal 500 μm	399.1 ± 78.9	402.5 ± 66.6
Nasal 1500 μm	358.6 ± 91.2	366.2 ± 76.9

All values are the mean ± standard deviation (μm).

The average ChTs at the temporal 500 μm, temporal 1500 μm, nasal 500 μm, and nasal 1500 μm points using SS- and SD-OCT were 407.8 ± 82.5 (range, 270.5 to 656.5 μm) and 409.1 ± 69.2 μm (range, 282 to 614.5 μm), 378.5 ± 87.0 (range, 201.5 to 637 μm) and 378.3 ± 77.6 μm (range, 208 to 620.5 μm), 399.1 ± 78.9 (range, 234.5 to 580 μm) and 402.5 ± 66.6 μm (range, 271 to 576.5 μm), and 358.6 ± 91.2 (range, 134.5 to 571.5 μm) and 366.2 ± 76.9 μm (169 to 546.5 μm), respectively. The average diameters of pachyvessel using SS- and SD-OCT were 281.76 ± 90.3 (range, 157 to 437 μm) and 278.9 ± 95.8 μm (range, 120 to 478 μm), and they were not significantly different (P = 0.772). In SS- and SD-OCT, a single choroidal cavern was observed in 10 and 12 eyes, and multiple choroidal caverns in 12 and 8 eyes, respectively, which did not show a significant difference (P = 0.770).

In repeated-measure ANOVA, measurement location showed a significant result as the main effect (P < 0.001). Other within-subjects such as OCT device, observer, and measurement order did not show a significant result as main effects (P = 0.067, P = 0.354, and P = 0.373, respectively).

### Interobserver and intraobserver repeatabilities of ChT measurements using SS-OCT and SD-OCT

The intraobserver ICCs of both observers were > 0.950 at every measured point using SS-OCT, which means high repeatability. The interobserver ICC of the subfoveal area, the temporal 500 μm, temporal 1500 μm, nasal 500 μm, and nasal 1500 μm points using SS-OCT was 0.929, 0.771, 0.864, 0.708, and 0.892, respectively. The intraobserver ICCs of both observers were > 0.800 using SD-OCT, which shows reasonable repeatability. However, the interobserver ICC of the subfoveal area, the temporal 500 μm, temporal 1500 μm, nasal 500 μm, and nasal 1500 μm points were 0.633, 0.657, 0.739, 0.689, and 0.767, respectively. Additionally, the intraobserver CR of both observers showed better repeatability in SS-OCT than SD-OCT, which was statistically significant in most areas (F-test, all P < 0.050 except nasal 1500 μm point in observer 2, P = 0.281) (Table 3). The interobserver CR also showed better repeatability in SS-OCT with statistically significance in some areas (subfovea, P = 0.014; temporal 500 μm, P = 0.619; temporal 1500 μm, P = 0.041; nasal 500 μm, P = 0.049; nasal 1500 μm, P = 0.569).

**Table 3:** Coefficient of repeatability (CR) of choroidal thickness measurements using swept source (SS) and spectral domain (SD) optical coherence tomography (OCT).

	Intraobserver 1 CR (μm, 95% CI)	Intraobserver 2 CR (μm, 95% CI)	Interobserver CR (μm, 95% CI)
SS-OCT			
Subfoveal	27.1 (24.5–29.7)	26.8 (24.2–29.3)	45.1 (40.8–49.4)
Temporal 500 μm	30.7 (27.8–33.6)	25.0 (22.6–27.4)	73.6 (66.6–80.7)
Temporal 1500 μm	31.8 (28.8–34.9)	34.8 (31.5–38.2)	72.0 (65.1–78.9)
Nasal 500 μm	35.2 (31.8–38.5)	29.0 (26.2–31.7)	91.1 (82.4–99.8)
Nasal 1500 μm	33.0 (29.9–36.2)	28.1 (25.5–30.8)	52.3 (47.3–57.3)
SD-OCT			
Subfoveal	42.3 (38.0–46.6)	43.8 (39.6–48.0)	71.2 (64.4–78.0)
Temporal 500 μm	46.8 (42.1–51.5)	48.4 (43.8–53.0)	78.3 (70.8–85.8)
Temporal 1500 μm	51.7 (45.9–57.5)	49.8 (45.0–54.5)	87.7 (79.3–96.0)
Nasal 500 μm	42.5 (39.1–45.9)	47.7 (43.2–52.3)	72.0 (65.1–78.9)
Nasal 1500 μm	43.9 (40.4–47.4)	30.8 (27.8–33.7)	61.1 (55.3–66.9)

CI, confidence interval.

In Bland-Altman plots, measurements using SD-OCT showed a larger scatter compared to those using SS-OCT (Fig 2).

**Fig 2:** Bland-Altman plots for agreement between two observers using swept source (SS) and spectral domain (SD) optical coherence tomography (OCT). The dashed lines show mean difference and 95% limits of agreement, and error bars mean 95% confidence intervals for limits of agreement. The spread points of SS-OCT were much smaller than those of SD-OCT.

### Interobserver reproducibility of ChT measurements using SS-OCT and SD-OCT in eyes with ChT ≥ 400 μm

To determine the reliability of ChT measurements in pachychoroid patients having thicker choroids, we analyzed 35 eyes with ChT ≥ 400 μm using two instruments. The ICCs of the subfoveal, temporal 500 μm, temporal 1500 μm, nasal 500 μm, and nasal 1500 μm points using SS-OCT were 0.880, 0.812, 0.842, 0.587, and 0.851, respectively. The ICC of the subfoveal area using SD-OCT was 0.499, and other areas also showed worse reproducibility than that of SS-OCT (Fig 3).

**Fig 3:** Bland-Altman plots for agreement between two observers using swept source (SS) and spectral domain (SD) (B) optical coherence tomography (OCT) in eyes with choroidal thickness ≥ 400 μm. The dashed lines show mean difference and 95% limits of agreement, and error bars mean 95% confidence intervals for limits of agreement. The differences in SD-OCT tended to be larger in patients with thicknesses ≥ 400 μm, whereas the differences in SS-OCT measurements were similar.

The interobserver CR of most areas also showed better repeatability in SS-OCT than SD-OCT (Table 4).

**Table 4:** Coefficients of repeatability of choroidal thickness measurements using swept source (SS) and spectral domain (SD) optical coherence tomography (OCT) in patients with choroidal thickness ≥ 400 μm (35 eyes).

	SS-OCT (95% CI)	SD-OCT (95% CI)
Subfoveal	48.4 (42.6–54.2)	95.2 (83.9–106.6)
Temporal 500 μm	74.7 (65.7–83.6)	89.9 (79.2–100.7)
Temporal 1500 μm	77.4 (68.1–86.7)	128.3 (113.0–143.7)
Nasal 500 μm	107.7 (94.8–120.6)	99.7 (87.7–111.6)
Nasal 1500 μm	59.0 (52.0–66.1)	78.6 (69.2–88.0)

CI, confidence interval.

### Interobserver reproducibility of ChT measurements using SS- and SD-OCT in eyes with subfoveal active lesions

To determine the reliability of ChT measurements in pachychoroid patients with subfoveal active lesions such as subretinal fluid, we analyzed 21 eyes with subfoveal lesions using the two instruments. The ICCs of the subfoveal, temporal 500 μm, temporal 1500 μm, nasal 500 μm, and nasal 1500 μm areas using SS-OCT were 0.925, 0.675, 0.834, 0.662, and 0.885, respectively. The ICCs using SD-OCT were 0.434, 0.400, 0.579, 0.726, and 0.766, respectively, indicating relatively low reproducibility (Fig 4).

**Fig 4:** Representative optical coherence tomography (OCT) images showing the difference in the clarity of the choroid-scleral boundary between swept source (SS) and spectral domain (SD) OCT. SS-OCT scan (A) and SD-OCT scan (B) of a patient with resolved central serous chorioretinopathy (CSC). The choroid-scleral boundary is observed more clearly in A than in B. SS-OCT scan (C) and SD-OCT scan (D) of a CSC patient with subretinal fluid (SRF). The choroid-scleral boundary of D is faint behind the SRF because of a shadow and hyperreflective layer within the choroid, whereas C shows a relatively clear choroid-scleral boundary.

The interobserver CR of all areas also showed better repeatability in SS-OCT than SD-OCT (Table 5).

**Table 5:** Coefficients of repeatability of choroidal thickness measurements using swept source (SS) and spectral domain (SD) optical coherence tomography (OCT) in patients with subfoveal active lesions (21 eyes).

	SS-OCT (95% CI)	SD-OCT (95% CI)
Subfoveal	44.5 (37.6–51.4)	100.1 (84.6–115.5)
Temporal 500 μm	93.7 (79.3–108.2)	99.2 (83.9–114.6)
Temporal 1500 μm	62.7 (53.0–72.4)	113.4 (95.9–130.9)
Nasal 500 μm	88.0 (74.4–101.5)	94.9 (80.2–109.5)
Nasal 1500 μm	58.5 (49.5–67.5)	67.3 (56.9–77.7)

CI, confidence interval.

## Discussion

With the advent of high-resolution SD-OCT, EDI has been widely used to image the choroidal structure. EDI obtains a good quality image of the choroid by moving the sensitivity curve at the sclera.[15] So previous studies have reported the measurement of the ChT in different pathologies using SD-OCT with EDI.[16–18] However, we encountered a considerable number of cases with pachychoroid diseases, in which SD-OCT with EDI could not measure the ChT because of an unclear choroid-scleral border. Whereas we could observe a relatively clear choroid-scleral border in those cases using SS-OCT. So we determined the comparability of ChT measurements using SS-OCT and SD-OCT in pachychoroid diseases to identify potential factors affecting the reliability of the measurements.

Several studies have assessed the comparability of ChT measurements using SS-OCT and SD-OCT in healthy subjects.[6–9, 19] Tan et al.[8] reported that subfoveal ChT measurements were comparable between SS-OCT and SD-OCT devices among normal eyes and eyes with retinal diseases such as age-related macular degeneration or diabetic maculopathy. Philip et al.[9] also reported that SD-OCT with EDI and SS-OCT, in young subjects with normal eyes, were interchangeable in their reliability in determining the ChT with a trend of ChT measurements being slightly thicker when measured using SD-OCT, which had limited clinical importance. In our study, the mean differences between 2 devices in each measurement location (subfovea, temporal 500 μm, temporal 1500 μm, nasal 500 μm, nasal 1500 μm) was 0.8 ± 32.1, -1.2 ± 46.3, 0.2 ± 43.6, -3.3 ± 42.5, and -7.6 ± 44.1 μm, respectively, which did not show a significant difference between 2 devices in a repeated-measure ANOVA (P = 0.063). Additionally, ChT measurements obtained using SD-OCT did not show significant thicker results than those acquired using SS-OCT. This difference may be the result of the different subjects examined in the two studies. Meanwhile, Matsuo et al.[19] reported that the ChT measurements were thicker using SS-OCT because the choroid-scleral border seen on SD-OCT scans may not be the true border. Synthetically, even though there is some possibility of a tendency to measure ChT thicker using any one device, the difference might be clinically insignificant.

Matsuo et al.[19] reported a high interobserver reproducibility of ChT measurements in healthy eyes using SS-OCT and SD-OCT, which were both over 0.990. Kong et al.[11] also reported that the ICC of subfoveal ChT measurements obtained using SD-OCT with EDI in healthy subjects, between two observers, was 0.995. In our study, the ICC of subfoveal ChT measurements in pachychoroid diseases using SS-OCT was 0.929, and the ICCs of other measured points were also reasonable, whereas the ICC of subfoveal ChT measurements made using SD-OCT was 0.633, and the ICCs of other points were lower than those obtained using SS-OCT. The interobserver CR using SS-OCT also showed higher repeatability in most areas than SD-OCT. Tan et al.[7] reported that there was a significant difference in the clarity of the choroid-scleral boundary between SS-OCT and SD-OCT in eyes with retinal diseases. In practice, in some cases, it was difficult to measure the ChT with SD-OCT because of an unclear choroid-scleral border. Although SD-OCT seemed sufficient to measure the ChT in healthy eyes, SS-OCT was more suitable for imaging the choroid of eyes with retinal diseases requiring observation of the choroidal structure in detail such as pachychoroid diseases.

In eyes with a ChT ≥ 400 μm, the difference of reproducibility between SS-OCT and SD-OCT was more definite. Whereas the CR and ICCs of SS-OCT were maintained to some degree, those of SD-OCT were remarkably decreased. Tan et al.[7] hypothesized that signal loss, artifacts, and shadows cast by the connective tissue between vessels might impair visualization of the choroid-scleral border more in SD-OCT than in SS-OCT in eyes with a thicker choroid. In patients with pachychoroid diseases, which have a ChT ≥ 400 μm in many cases, it might be difficult to accurately measure the ChT using SD-OCT. However, ChT may not be the only factor affecting the image quality of the choroid-scleral border, because it was observed relatively clearly in normal eyes with a thick choroid.

The image quality and clarity of the choroid also seemed to be affected by the presence of pathologies, such as subretinal fluid, drusen, or a hard exudate. In eyes with subfoveal active lesions such as subretinal fluid, the subfoveal CR and ICC of SD-OCT showed low repeatability compared to that of SS-OCT. The choroid-scleral boundary looked faint or absent because of the shadow appearing just behind the lesion. A previous study reported that better penetration through media opacities is one of the advantages of the long-wavelength SS-OCT device.[20] The 1050 nm OCT system penetrates more deeply, and consequently has high sensitivity for the posterior choroidal boundary and the sclera, which allows better visualization of the chorioscleral interface, whereas the 840 nm SD-OCT system does not penetrate as deeply and has a higher portion of scattered light.[9] In pachychoroid diseases, which have both conditions of thick choroids with a high probability of subfoveal lesions, SS-OCT is therefore more appropriate to observe and follow-up the choroidal structure in detail.

Our study showed CRs more than 100 μm in some locations using the SD-OCT in patients with ChT ≥ 400 μm and subfoveal lesions. This was high CRs comparing with other studies for healthy subjects, which was typically in the range of less than 30 μm.[21, 22] The CRs using the SS-OCT in these groups was also higher than that of previous studies. These might result from the thick and relatively uneven posterior choroidal boundary besides the faint images. Whereas normal subjects have relatively even and flat choroid, patients in these groups have uneven and different choroidal thickness according to the location because of pachyvessels. When measuring the choroidal thickness several times according to the location, there might be a slight difference in measurement location at each measurement, which might affect bigger differences between measurements in these groups than normal subjects.

### Study limitations and strengths

Our study had several limitations. First, we used manual segmentation because these 2 OCT devices could not segment the choroidal layer automatically, which may have included uncontrolled bias among examiners. However, the observers were well-trained and experienced, and the intraobserver repeatability was relatively high on each device. Second, we evaluated the specific scanning protocol of each SD-OCT and SS-OCT instrument, but it is uncertain whether our observations can be adjusted to other OCT devices or other scanning protocols. Third, the points of thickness measurement using each device might be slightly different because of the difference in the resolution of 2 devices.

The strength of our study was that we compared SS-OCT and SD-OCT among patients with pachychoroid diseases, in which a detailed observation of the choroidal structure is needed. To the best of our knowledge, a comparison of the two devices in pachychoroid diseases has not been previously reported. Additionally, we determined the low repeatability of ChT measurements obtained using SD-OCT in patients with ChT ≥ 400 μm, and assessed the impact of subfoveal lesions, such as subretinal fluid, among pachychoroid patients. We also performed the OCT scans on different devices consecutively, within a few minutes of each other, to minimize the potential effects of diurnal variation.

In conclusion, although the ChT measurements were comparable between the SS-OCT and SD-OCT devices when measuring patients with pachychoroid diseases, SD-OCT had limitations providing accurate and clear images in patients with thicker choroids and subfoveal active lesions. SS-OCT would be therefore more suitable for observation and follow-up of choroidal structures in patients with pachychoroid diseases.

## Supporting information

S1 Data (XLSX)
